This article has been retracted.

# The Relevance of Virtual-Assisted Early Childhood Education and Occupational Psychotherapy Based on Emotional Interaction

**DOI:** 10.1155/2022/2785987

**Published:** 2022-07-14

**Authors:** Dingran Qie

**Affiliations:** Graduate Schools, Keimyung University, Daegu 42601, Republic of Korea

## Abstract

This paper presents an in-depth study and analysis of the relevance of early childhood education to occupational psychotherapy using a virtual-assisted affective interaction approach. Starting from the educational theory of interactive cognitive psychology, the theoretical basis for parent-child picture book education for interactive learning is explored, as well as the theoretical development after the introduction of AR technology. Firstly, the analysis of young children's emotions involves massive image processing, and the use of cloud computing architecture leads to high latency, while young children's safety is a latency-sensitive service. Secondly, face recognition accuracy based on static images is not high due to problems such as inconspicuous facial features of toddlers and low-quality kindergarten surveillance videos. In this paper, a face identity correction model based on location features is proposed and the superiority of the model is demonstrated through experiments. Finally, this paper analyzes and mines the emotional data of young children. The level of kindergarten teachers' awareness of early childhood mental health education generally showed an upward trend as their titles rose, and there were significant differences in the seven dimensions of early childhood mental health, the purpose and meaning of early childhood mental health education, implementers, targets, content, pathways, and effects; significant differences existed between teachers of different kindergarten natures, and there were significant differences in the purpose and meaning of early childhood mental health education, implementers, targets, content, pathways, effects, and mental health education for young children. Therefore, this paper proposes a face identity correction model based on position information, which considers both the correlation between pixel values in the spatial domain and the correlation between frames in the temporal domain. This paper has developed an emotion analysis system for kindergartens and put it into use in kindergartens to meet the needs of monitoring the safety of young children and evaluating early childhood education and has received good feedback from users, demonstrating the effectiveness of the system.

## 1. Introduction

Emotional interaction cannot be achieved without the technical means of artificial intelligence. For more than two decades, AI researchers have been trying to give machines the cognitive ability to recognise, interpret, and express emotions [1]. By correlating, analyzing, and reconstructing data containing emotional information from different scenarios, artificial intelligence technologies eventually transform the data into abstract thoughts that computers can understand, thereby simulating human emotional cognition and decision-making processes; i.e., the emotional interaction process uses the user's modal data to recognise the user's emotional state, uses the feedback from the emotional recognition to model emotions based on cognitive analysis, and guides the interaction behavior. Therefore, the emotion recognition process and the emotion modeling process are the two most important steps of affective interaction. However, due to the complex nature of multimodal data distribution and the problem of personalization between different users, there are limitations in the study of personalized affective interactions based on multimodal data, so there is an urgent need to investigate the association and integration of modal data in conjunction with learning models to improve the performance of affective interactions around application scenarios [2]. In this paper, this method is used for training. The garden teachers provide sample photos of each child and mark their identities and fine-tune the official open-source trained FaceNet model. From previous research on the ways of professional growth of kindergarten teachers, teachers' professional growth is mainly based on in-service training and garden-based on-site teaching and research, both of which have achieved significant results in promoting kindergarten teachers' professional development but also have many problems. Past studies have looked at different groups, such as rural teachers and core teachers, from both macro and micro perspectives and at the micro level, mainly from the various aspects of training to examine the problems faced by teachers in the training process.

Starting from the educational theory of interactive cognitive psychology and combining the display and interaction methods of AR technology, the parent-child picture book reading and parent-child picture book game are analyzed and the activity organization model, interaction means, and content are redesigned. By analyzing the traditional parent-child picture book reading model, the content, approach, and process of parent-child reading in the AR environment are proposed, and a new AR interaction for parent-child reading is constructed. As the safety and education of young children are receiving increased attention, many visual sensors are installed in kindergartens to monitor children, generating a large amount of image data daily. A key technical issue is the detection of unusual events and responding to them quickly. Unusual events in kindergartens can range from personal to environmental causes [3]. A common feature of these unusual events is that children often express negative emotions, such as anger, sadness, and fear. The processing of images containing negative emotions is therefore latency-sensitive for kindergartens and requires a system that can analyze children's emotions in real time and notify the relevant personnel with less latency. Managing and processing this image data in the cloud can lead to increased latency, reducing the efficiency of network traffic management and computational processing.

Psychological normality and psychological abnormality are opposing concepts, with psychological abnormality usually referring to a psychological state with a typical mental disorder [4]. Mental health, on the other hand, and mental ill-health belong to a pair of concepts within the range of psychological normality. Mental health generally signifies an individual with a relatively stable internal psychological environment, with good self-awareness and the ability to adapt to the environment, and exhibiting socially acceptable emotional and behavioral states. Different scholars have different definitions of mental health. The applications related to emotion data of young children are still in the initial exploration stage, and scholars are enthusiastic about emotion recognition, but how to use the experimental data generated by emotion recognition for further data analysis and to generate a positive impact on real life is a major difficulty of current research. Therefore, there is a need to mine and analyze the data on young children's emotions and to quantify and visualize the data according to parents' needs for the safety and education of young children. It can make up for the cognitive scene at the scale of people's observation and reduce the macro-scale world to the scale of the current field of vision. When the system identifies negative emotions in children, kindergartens should pay more attention to them; and based on the analysis of the emotional data of individual children and teachers, early childhood education can be evaluated, providing a pedagogical reference for schools and parents.

## 2. Related Works

Psychotherapy originated from the psychoanalysis founded by Sigmund Freud in the late 19th century. As a medical model, psychotherapy is aimed at relieving patients of their symptoms and suffering. Psychotherapy is a process whereby a trained therapist uses the relevant theories and techniques of psychology to help patients eliminate and alleviate serious psychological problems and disorders, promote the healthy and harmonious development of their personality, and restore their mental health, based on the establishment of a good therapeutic relationship [5]. In the early days, people equated mental health education with psychotherapy, to provide help to a small number of people with serious psychological problems and disorders. Psychological counselling is the process of establishing a certain interpersonal relationship with the client with the help of language, text, and other media and using psychological theories and techniques to help the client eliminate psychological problems and obstacles and improve his or her mental health [6]. The goal of counselling is to correct the psychological disturbances and mild to moderate disorders of adaptation and development that occur in normal people in social life. In the medium term, people equate mental health education with counselling, and counselling is the transitional link between psychotherapy and psychological counselling. Counselling is the result of the gradual development of psychological counselling in schools. Counselling has a broader meaning and can be equated with mental health education in most cases [7]. The game design that is adapted to the physical and mental development of young children promotes the smooth progress of the game. Mental health education is the inevitable result of the further development of counselling, and mental health education becomes an integral part of the quality education system. It can thus be seen that the purpose and meaning of mental health education have undergone a process of transformation from a medical model to a pedagogical model and from remedial to developmental goals.

Ismail and others believed that the physical health of young children was as important as their mental health, and they were the first to advocate the development of mental health education programmed for young children in kindergartens [8]. Javaid and Haleem were the first to study kindergarten mental health education programmers, introducing the American mental health education programmed “Bibi and Friends” to a kindergarten in Shanghai [9]. Papanastasiou et al. proposed a method of using physiological signals to identify emotions [10]. However, due to the high density of people in kindergartens, emotion recognition through video and audio can be noisy; wearing a microphone for each child is costly; and using physiological signals for emotion recognition usually requires the child to wear multiple biosensors, such as ECG receivers or respiratory sensors, which are not suitable for long-term monitoring [11]. Farr et al. use convolutional neural networks to extract features from GSR signals and use an end-to-end approach for emotion state recognition, achieving 85% recognition rates on the database [12].

Since people can communicate and cooperate through the expression of human emotional states, much work and research have been done to try to give computers the ability to emotionally interact with humans and machines [13]. The application areas of affective interaction are in a variety of fields such as elderly care, cognitive rehabilitation, and intelligent education. The content of the game should be in line with the cognition of children and remember not to exceed the cognition of children. In intelligent education, for example, effective interaction can be used to motivate learning, adjust teaching strategies according to affective states, and provide personalized teaching services. This paper proposes a combined cloud-edge system architecture and an optimization algorithm for prioritizing scheduling based on job content, reducing the overall latency of the system, i.e., the latency from the edge server acquiring the images to the cloud server recognizing and analyzing the images and making the final visual display. Based on the business scenario of the kindergarten, we propose a system architecture and detailed deployment plan that combines edge computing and cloud computing to reduce the latency problem under massive data. A priority scheduling algorithm is designed based on the results of emotion detection of children, which increases the throughput of abnormal data processing per unit time and reduces the overall latency of abnormal event response.

## 3. An Analysis of the Relevance of an Emotionally Interactive Integration of Virtual Support Methods for Early Childhood Education and Occupational Psychotherapy

### 3.1. Design of a Virtual Aid for Emotional Interaction Integration

Emotion is the feeling of something based on its satisfaction with one's needs, and interaction means communicating with each other. The term emotional interaction is mostly found in interaction design. Interaction design refers to the content and structure of communication between two or more interacting individuals to collaborate to achieve a specific goal. Its design kernel is concerned with human-centred user needs. Interaction design usually places more emphasis on human-computer interaction. In this paper, however, interaction is primarily invoked in its original sense, as communication and interaction [14]. The emotional interaction mentioned in this paper highlights the user's communication and interaction with the product on an emotional level, with an emphasis on personal interaction. Its fundamental purpose is the same as interaction design, which is to meet the spiritual needs of users and to enhance the emotional design experience to serve people.

Emotion is a unique human cognition with social needs, which is relatively stable. Based on the premise of emotional cognition, designing interactive products that can elicit positive responses from users and meet their emotional needs is the completion of the construction process of emotional interaction. The definition of emotional interaction should be explored from the perspective of both the subject and the object. The subject applies emotion to the object after generating an emotional appeal, and the object generates a corresponding emotion after receiving the subject's emotion and responding, the identity of both the subject and the object is transformed, completing an interaction. The relationship between emotion and interaction complements each other, with interaction being how the product conveys emotion to the audience, and emotion increasing the variety of interaction, both of which support each other.

Augmented reality is an emerging form of experience in which augmented content seamlessly integrates real-world information with virtual-world information, allowing things that cannot be experienced in the real world to be displayed in the real world through AR technology [15]. However, depending on the feature fusion method in the form of single-modal concatenation, the semantic correlation between modalities is not considered, which makes it impossible to guarantee the semantic consistency between the modal features of the final input recognition model. These virtual objects are superimposed multiple times and are perceived by the human senses of sight, touch, hearing, and taste. Augmented reality technology encompasses interaction techniques such as real-time interaction, real-time tracking, real-time registration, a fusion of reality and reality, and the display of virtual and real information. Hardware-based interaction and computer vision-based interaction are two of the most popular augmented reality interaction techniques. Hardware-based interaction requires tracking devices, such as AR glasses and physical wearable devices. Therefore, this paper considers personalized emotional interaction, including not only the personalized emotion recognition process but also the emotion modeling process under different preference settings. The emotion modeling process considers the evolution of the temporal dimension and the transfer of emotional states based on cognitive reevaluation capabilities to achieve positive emotional interactions. Behavioral decisions are the output of a joint cognitive-emotional interaction, rather than being based on a simple rule mapping.

As shown in Figure 1, the closed-loop process of emotional interaction in this paper includes sensor input, emotion perception (emotion recognition), emotion modeling, and behavioral decision-making. The user's modal data is input to the smart device through sensors, and the smart device can sense the user's emotional state now based on the feature processing and recognition process. Based on the user's emotional state and interaction behavior, the smart device can generate feedback behavior and emotional expressions through emotional awareness decisions.

Due to the different sources of modal data, the form of sentiment information implied by each modality is different. Therefore, the feature extraction process, which corresponds to the emotion recognition process, needs to consider the characteristics of each modal data, to transform the original data form into effective emotion features and improve the ability of features to characterize the semantics of emotion. Thus, the original data form is transformed into effective emotional features, and the ability of features to represent emotional semantics is improved. However, feature fusion in the form of single-modal concatenation does not consider the semantic correlation between the modalities, which makes it impossible to guarantee the semantic consistency between the modal feature input to the final recognition model [16]. In this paper, we propose a multimodal feature processing method that incorporates sentiment semantic analysis to improve the ability of multimodal features to characterize sentiment semantics.

Children of different ages have different physical and mental developmental characteristics, so the design of AR parent-child games should take into full consideration the age characteristics of children, and what is appropriate is the best. Firstly, the difficulty level should be set to suit, not too high for children to complete, and not too easy to be challenging; secondly, the game content should be in line with children's cognition and not beyond their cognitive range. A game design that is appropriate to the child's physical and mental development promotes smooth play.

Therefore, this paper considers personalized emotional interaction, including not only the personalized emotion recognition process but also the emotion modeling process under different preference settings. In traditional listening and sensory reading, although parents and children can follow a certain plan and complete a certain amount of reading in a certain amount of time, the reading process is often not as engaging as it could be due to the parents' inability to use emotionally enriching language and the lack of realistic and visible images of the characters in the picture book.

Professional workers without full professional education or training are influenced by contextual activities and acquire problem-solving skills through interactions with others, the environment, etc. Further research has found that knowledge needs to be presented through real situations and concrete applications and that learning needs to occur in a specific cultural environment to be effective [17]. AR parent-child games, which can apply modern modeling, 3D simulation, and multimodal interaction technologies to create virtual learning situations, can compensate for the cognitive scenarios at the scale of people's observations, reducing the macro-scale world to the scale of current vision.

Children are passive listeners in the reading process, unable to concentrate on the boring story, and unable to appreciate the charm of the picture book nor to exercise their observation and thinking skills, thus failing to achieve the desired reading effect.

In practical application scenarios, face recognition usually encounters a situation where the sample dataset is too small; i.e., the number of training samples is much smaller than the number of faces to be recognized. This problem is often solved by migration learning, where a model trained on one problem is adapted to a new problem with simple adjustments. Hardware-based interaction requires tracking devices, such as AR glasses and somatosensory wearable devices. In this paper, we use this approach for training, where the teacher provides a sample photo of each child and marks the identity and fine-tunes the official open-source trained FaceNet model. However, since the recognition target is a toddler, the face is smaller and less distinct than that of an adult, and the FaceNet palace-side training model is trained using the VGGFace dataset, which has a very small proportion of toddler pictures, which will affect the final recognition accuracy. As shown in Table 1, the recognition results of a class of 12 children in a 30-minute session within the kindergarten were counted, with 58% of the children recognized with less than 80% accuracy and overall average recognition accuracy of approximately 63%, and one child with ID 16 who was absent that day was mistakenly recognized once. Such face recognition accuracy is not yet at a level where it can be applied and will affect the final sentiment sequence analysis.

To this end, this paper proposes two solutions to improve the above face recognition results. One is to design an annotation system to enhance the data from the perspective of the training sample, i.e., the dataset. Since there are significant differences in lighting, pixel size, and viewing angle between the samples provided by the school and the images captured by the sensors, the annotation system can be used to filter homologous samples from all angles of the children to be added to the training. Secondly, the secondary recognition is combined with the location information of the toddler to correct the face identity [18]. The object generates corresponding emotions after receiving the subject's emotion, and after the response, the identities of the subject and the object are transformed to complete an interaction. Most of the current face recognition is through static image recognition, which only learns the features between the pixel values in the image while ignoring the motion features based on the location information. The former can describe the appearance of the object, while the latter describes the motion of the object in the video. Therefore, this paper proposes a face identity correction model based on location information, considering both the correlation between pixel values in the spatial domain and the correlation between frames in the temporal domain.

Early childhood is a time of rapid intellectual and creative development and is at its best when it can be nurtured through a variety of literary and artistic activities. The formation and development of young children's creativity can be achieved by nurturing their curiosity and creative imagination in the preschool educator's class, as shown in Figure 2. Because young children's curiosity is the starting point for the development of creativity, an individual with a high level of creativity must have a high level of curiosity. A good visual environment and atmosphere are of great importance to children's creative imagination.

The dynamic nature of graphics is the ability of graphics to change their form over time, a new characteristic of visual communication design that has emerged in response to advances in technology [19]. In the traditional field of visual communication design, the focus is on the static visual representation of a graphic medium; making graphics dynamic is a way of creating a visual symbol based on moving image material on top of the graphic design. In the early stages of observation, the subject's emotions and interests can easily influence the state of observation, as can changes in the object to varying degrees.

### 3.2. Analysis of the Relevance of Early Childhood Education to Occupational Psychotherapy

All eight public kindergartens have easy access to the Internet, achieving full coverage of the campus network, while the situation in private kindergartens is more difficult, with 11 kindergartens having easy access to the Internet and five kindergartens not having easy access to the Internet, which is a fundamental constraint to the professional growth of teachers using digital resources [20]. Its fundamental purpose is no different from interaction design. It is also to meet the spiritual needs of users, improve the emotional design experience, and serve people. In general, the public kindergartens have an absolute advantage in terms of the configuration of infrastructure and equipment, which facilitates teachers' easy access to digital resources for self-directed learning, and teachers in public kindergartens are more willing to invest in digital equipment in terms of the number of laptops they own individually or at home. Both the individual and the kindergarten's digital facilities are not conducive to their use of digital resources. In general, however, the infrastructure of kindergartens is gradually being optimised, but further improvements are needed.

To support the experiment, webcams were installed in the classrooms to obtain image data from 10 different classes within the kindergarten. During sessions lasting 30 minutes, the cameras captured the children's facial expressions every 10 seconds [21]. The different children were first identified, and each child was assigned an ID; then, the emotions of each face in the identified images were stored in a database and this emotional data formed the basis for data mining.

The dataset is based on a collection of images from two lessons in each of two classes selected from the kindergarten, with the emotional recognition of each face in each image counted as one piece of data, with a total of 14,049 pieces of data, including 38 children with different identity IDs, covering seven emotions: anger, contempt, disgust, happiness, calmness, sadness, and surprise. According to the timing of the video, four sessions were involved, each lasting 30 minutes. As shown in Figure 3, the “calm” emotion accounted for more than 90% of all the emotion data. Have good self-awareness and environmental adaptability, and demonstrate socially acceptable emotional and behavioral states. At the same time, happiness, sadness, and surprise accounted for an appropriate proportion. However, anger, contempt, and disgust were rarely encountered. In a kindergarten setting, children are most attentive and calm, with a few instances of mood swings due to interactions with the teacher or influences from the surrounding environment, and these noncalm emotions are the ones that deserve to be analyzed.

Teachers' perceptions of early childhood mental health education showed significant differences in these five significantly different dimensions on the boundary between college and bachelor's degree, showing that kindergarten teachers trained by preschool education majors at the bachelor's degree level and above have a higher level of awareness of early childhood mental health education [22]. The differences in the three dimensions of perceptions of early childhood mental health, the effectiveness of early childhood mental health education, and the relationship between early childhood mental health education and moral education were not significant.

This may be because the sample size for this title is only one, which is not statistically significant. Anomalies in kindergarten can range from personal to environmental causes. The mean scores of teachers with senior titles were significantly higher than the scores of teachers at other levels. There was no significant difference between the scores of teachers with the title of Level 1 and Level 2 in their views on early childhood mental health education, and there was a significant difference between teachers with the title of Level 3 and teachers with the titles of Level 1 and Level 2 in their views on early childhood mental health education. In summary, the level of kindergarten teachers' awareness of early childhood mental health education showed an upward trend as their job titles rose. The decreasing trend in scores between nonparticipating teachers to Level 3 teachers and Koran teachers to full senior teachers may be due to the small sample size, resulting in lower overall scores, as shown in Figure 4.

As shown in Figure 4, the correlation between affective states and behavioral decisions is usually lower than the correlation between motivation and behavioral decisions. Where the correlation coefficient between motivation and behavioral decision-making is low, the correlation coefficient between affective state and behavioral decision-making is usually higher than in the rest of the cases. This demonstrates that different subjects elicit different control factors for behavioral decision-making [23]. The robot can make behavioral decisions that fit the different distributions based on the behavioral data fed back by different subjects, which is one of the goals of personalized interaction. Regarding the effect of motivation on emotion, a correlation coefficient greater than 0.4 can be seen, which means that motivation has an arousing effect on emotion.

By comparing the scores of teachers with different job titles on each dimension, we found that there were significant differences in the knowledge of teachers with different job titles on the seven dimensions of early childhood mental health, the purpose and meaning of early childhood mental health education, the implementer, the target, the content, the ways, and the effects. Given that the number of senior teachers is limited and not representative, no specific analysis is conducted in this paper. A large amount of image data is generated every day. A key technical issue is detecting anomalous events and responding quickly to them. In general, there is a downward trend in the scores of teachers' perceptions of education from high-ranking teachers to nonparticipating teachers, indicating that the higher the teacher's title, the higher the level of awareness of mental health education for young children.

## 4. Analysis of Results

### 4.1. Performance Results of the Emotional Interaction Fusion Virtual Assistance Method

The samples collected in Experiment 1 form the initial training set for the validation of this section, and the feature processing and recognition model algorithms proposed in this paper are integrated into the personalized emotional interaction learning platform. The integration was mainly performed in Experiment 2; specifically, the platform captured the subject's peripheral physiological signals and facial expressions through the wearable wristband and camera; the 16-frame video signal was processed by the C3D algorithm and the DBN and manually extracted features based on the peripheral physiological signals; the features were further processed using the trained feature processing module in the training set and input to the T-SVR model for emotion recognition. The final recognition results were compared with the subject's self-rated affective state in the corresponding phase of the experiment, assessed using the CCC metric.

Figure 5 shows the results of the comparison of the recognition algorithms based on the interaction dataset, with the recognition results without semantic analysis fusion being lower than those with semantic analysis feature processing. The most significant improvement in recognition results for the support vector regression model was achieved by semantic fusion. This demonstrates that semantic analysis fusion can further process the initial features and extract key information to assist the supervised learning-based recognition model in finding patterns. As SVR, ridge regression, and lasso regression cannot be trained to produce effective recognition models based on the full training set, all three are based on subject-related training methods. A comparison of the recognition algorithms shows that the proposed T-SVR achieves the best recognition rate. As the dataset was collected from an interactive experiment with 40 individuals, each subject contains an average of 60 samples, which is in line with the characteristics of a small sample dataset. Transduction learning can build local training models and effectively solve problems such as poor generalisation ability of small sample datasets.

The first phase of the experiment corresponds to an ablation experiment of emotion modeling, which can subtract the effect of recognition effects on emotion modeling. At the micro level, it mainly starts from all aspects of training to examine the problems faced by teachers in the training process. The data from the human-machine affective interaction experiment in Experiment 1 were analyzed to measure the effects of different affective-cognitive collaboration model parameters on learning outcomes. As subjects' academic emotions and scores were influenced by a variety of factors, the mean and variance of the data from Experiment 1 and Experiment 2 were observed to fluctuate using statistical analysis. In Experiment 2, the mean values of academic mood and scores were slightly lower than in Experiment 1, with an average variation of 9%.

Due to the small average variation, it is shown that the results of emotion recognition as an external incentive to engage in affective interaction can achieve effective results. Together with the analysis of learning outcomes, the overall effectiveness of personalized affective interaction based on multimodal affective semantic analysis was verified, as shown in Figure 6.

After clustering and analyzing the emotions of the children in the programme, two children with abnormal emotions were identified, and after video verification, they did have abnormal emotions due to a change in the teacher's teaching style, while they were more active and focused in the interactive teaching. This helped the school and parents to identify the children's interests. From the perspective of past research, it has been carried out for different groups, such as rural teachers and key teachers, from two perspectives, macro and micro. Overall, it is normal and common for most children to show curiosity and delight in new things in the classroom. However, there are also a few children in each class who show extreme negative emotions or dramatic mood swings. These exceptional cases need to be noticed and helped promptly. The benefits of detecting and analyzing emotions in real time can therefore be demonstrated. Teachers can use the results of these data analyses to see whether the curriculum fits the cognitive habits of the children and whether the children are willing to accept this approach to education.

### 4.2. Relevance Analysis

The *t*-test showed that the difference between public and private kindergarten teachers was significant in their perceptions of the seven dimensions of the purpose and meaning of mental health education for young children, implementers, targets, content, approaches, effects, and the relationship between mental health education for young children and moral education and highly significant in their perceptions of the two dimensions of the targets and approaches of mental health education for young children, while there is difference in their perceptions. The differences were not significant in the perceptions of the seven dimensions of mental health education. In general, both public and private schools scored the highest on the dimension of mental health and the lowest on the dimension of the relationship between mental health education and moral education.

Most teachers have a shallow understanding of the various dimensions of mental health education for young children, and their understanding of the specific content of each dimension is blurred and one-sided. For example, in terms of teachers' understanding of the purpose and meaning of mental health education for young children, there are doubts as to whether “solving young children's psychological problems” should be included in the objectives of mental health education for young children; some teachers simply equate the means of mental health education for young children with psychological tests or counselling activities. Most teachers are aware of the need for tripartite cooperation among kindergartens, families, and the community in early childhood mental health education, but their understanding of specific approaches to early childhood mental health education is one-sided and ambiguous. These two methods have achieved remarkable results in promoting the professional development of kindergarten teachers, but there are also many problems. This may be because kindergartens do not pay enough attention to early childhood mental health education and have not conducted any teaching activities or training specifically for teachers, as shown in Figure 7.

In all aspects of teachers' needs, teachers have a predominance of visual and digital graphic resources in the presentation of digital resources; a tendency to use professional applications to access digital resources; the highest demand for the function of communication, sharing, and discussion of digital resources; and higher demand from teachers for the function of interpersonal interaction, which is currently the weak point of digital resources. In the management analysis of the class, this paper focuses on quality assessment and safety testing based on the number of times each type of emotion occurs.

In terms of the content of digital resources, teachers have the highest demand for professional knowledge and teaching knowledge, showing a tendency towards pragmatism, and a lower level of demand for classroom management and general knowledge, based on the fact that classroom management teachers are more inclined to use garden-based teaching and research or one-to-one support, with the old leading the new, to gain growth, and this content is generally reflected by teachers as easy to get started and easy to solve. The general knowledge is not very practical for teachers and is difficult to demonstrate through learning, so kindergarten teachers have the lowest level of need and generally report that they do not need this knowledge.

The emotional interaction process uses the user's modal data to realize the recognition of the user's emotional state and uses the feedback information of emotion recognition to perform emotional modeling based on cognitive analysis. The number of children experiencing negative emotions at any one time is counted, and safety alerts are given when the threshold is exceeded; the number and proportion of children experiencing negative emotions are counted, and classes are classified as priority classes when the number of children experiencing severe emotional fluctuations exceeds the average for each class.

Based on the above assessment, a classroom management assessment was conducted for one classroom and during the afternoon, the system collected negative emotions from some children and prompted notification of this. The emotion data identified by the system was plotted, as shown in Figure 8, with the meaning of the emotion represented by each color on the right-hand side, and the previously detected emotions of each child are also shown together for comparison purposes. As can be seen from the graph, as many as six children were experiencing negative emotions of sadness at the same time at this moment.

The above analysis proves the usefulness of the system, which allows for timely handling and notification when abnormalities are detected, effectively preventing the occurrence of hazards. In addition, the system can be used as a yardstick to measure each class. Through continuous evaluation in stages, trends in the management of each class can be identified, the rationality and effectiveness of the management style can be objectively assessed, and competition can be formed within each class to help improve the quality of class management and teaching.

## 5. Conclusion

This paper focuses on the current hot topic of early childhood safety and education, through face recognition and emotion recognition of young children, to grasp the emotional dynamics of young children in real-time and quantify the emotional data for in-depth analysis. Emotions provide the most direct way to understand children, and real-time monitoring of abnormal emotions can improve the safety of children in kindergartens. The mining of emotional data also provides a great reference for assessing children's learning, classroom management, and the effectiveness of the curriculum. And the superiority of this model is proved by experiments. All of this facilitates managers to have an accurate direction of children's growth and helps in decision-making for early childhood education and teaching and children's growth. The importance attached to early childhood mental health education has deepened; there are some ambiguity and one-sidedness in the specific understanding of early childhood mental health education and confusion between early childhood mental health education and moral education. Early childhood teachers' views on early childhood mental health education are influenced by five factors: teachers themselves, kindergartens, educational administration, society, and theory. Specifically, teachers' preservice learning backgrounds, teachers' experiences, kindergartens' educational concepts, teaching and research activities, teacher training, requirements of administrative departments, requirements of social development, and theoretical construction are all different. The teachers' views on early childhood mental health education are influenced to different degrees.

## Figures and Tables

**Figure 1:** The closed-loop process of emotional interaction.

**Figure 2:** Virtual-aided design framework.

**Figure 3:** Statistical overview of the emotion dataset.

**Figure 4:** Correlation coefficients for different configurations.

**Figure 5:** Comparison of results between recognition algorithms.

**Figure 6:** Normalization results and clustering categories for young children's characteristics.

**Figure 7:** Situation by dimension.

**Figure 8:** Emotional data correlation demonstration.

**Table 1:** Initial face recognition accuracy statistics.

Toddler ID	Total faces	Accuracy
48	173	99.3
47	230	95
46	379	96.7
35	278	96.3
14	229	97.6
28	385	96.6
41	377	96.2

## Data Availability

The data used to support the findings of this study are available from the corresponding author upon request.

## References

[1] Ghanouni P., Jarus T., Zwicker J. G., Lucyshyn J., Mow K., Ledingham A. (2019). Social stories for children with autism spectrum disorder: validating the content of a virtual reality program. *Journal of Autism and Developmental Disorders*.

[2] Lee I. J. (2021). Kinect-for-windows with augmented reality in an interactive roleplay system for children with an autism spectrum disorder. *Interactive Learning Environments*.

[3] Cahill S. M., Egan B. E., Seber J. (2020). Activity-and occupation-based interventions to support mental health, positive behavior, and social participation for children and youth: a systematic review. *The American Journal of Occupational Therapy*.

[4] Lu A., Chan S., Cai Y., Huang L., Nay Z. T., Goei S. L. (2018). Learning through VR gaming with virtual pink dolphins for children with ASD. *Interactive Learning Environments*.

[5] Huang Y. C., Backman S. J., Backman K. F., McGuire F. A., Moore D. W. (2019). An investigation of motivation and experience in virtual learning environments: a self-determination theory. *Education and Information Technologies*.

[6] Marino F., Chilà P., Sfrazzetto S. T. (2020). Outcomes of a robot-assisted social-emotional understanding intervention for young children with autism spectrum disorders. *Journal of Autism and Developmental Disorders*.

[7] Huang C. L., Luo Y. F., Yang S. C., Lu C. M., Chen A. S. (2020). Influence of students’ learning style, sense of presence, and cognitive load on learning outcomes in an immersive virtual reality learning environment. *Journal of Educational Computing Research*.

[8] Ismail L. I., Verhoeven T., Dambre J., Wyffels F. (2019). Leveraging robotics research for children with autism: a review. *International Journal of Social Robotics*.

[9] Javaid M., Haleem A. (2020). Virtual reality applications toward medical field. *Clinical Epidemiology and Global Health*.

[10] Papanastasiou G., Drigas A., Skianis C., Lytras M., Papanastasiou E. (2019). Virtual and augmented reality effects on K-12, higher and tertiary education students’ twenty-first century skills. *Virtual Reality*.

[11] Makransky G., Petersen G. B. (2021). The cognitive affective model of immersive learning (CAMIL): a theoretical research-based model of learning in immersive virtual reality. *Educational Psychology Review*.

[12] Farr W. J., Green D., Bremner S. (2021). Feasibility of a randomised controlled trial to evaluate home-based virtual reality therapy in children with cerebral palsy. *Disability and Rehabilitation*.

[13] Grabowski K., Rynkiewicz A., Lassalle A. (2019). Emotional expression in psychiatric conditions: new technology for clinicians. *Psychiatry and Clinical Neurosciences*.

[14] Crawford A., Vaughn K. A., Guttentag C. L., Varghese C., Oh Y., Zucker T. A. (2021). “Doing What I can, but I got no Magic Wand:” A Snapshot of Early Childhood Educator Experiences and Efforts to Ensure Quality During the COVID-19 Pandemic. *Early Childhood Education Journal*.

[15] Zhao H., Swanson A. R., Weitlauf A. S., Warren Z. E., Sarkar N. (2018). Hand-in-hand: a communication-enhancement collaborative virtual reality system for promoting social interaction in children with autism spectrum disorders. *IEEE transactions on human-machine systems*.

[16] Chang C. Y., Sung H. Y., Guo J. L., Chang B. Y., Kuo F. R. (2022). Effects of spherical video-based virtual reality on nursing students’ learning performance in childbirth education training. *Interactive Learning Environments*.

[17] Lang S. N., Jeon L., Sproat E. B., Brothers B. E., Buettner C. K. (2020). Social emotional learning for teachers (SELF-T): a short-term, online intervention to increase early childhood educators’ resilience. *Early Education and Development*.

[18] Hilty D. M., Randhawa K., Maheu M. M. (2020). A review of telepresence, virtual reality, and augmented reality applied to clinical care. *Journal of Technology in Behavioral Science*.

[19] Miller I. T., Wiederhold B. K., Miller C. S., Wiederhold M. D. (2020). Virtual reality air travel training with children on the autism spectrum: a preliminary report. *Cyberpsychology, Behavior and Social Networking*.

[20] Walker G., Weidenbenner J. V. (2019). Social and emotional learning in the age of virtual play: technology, empathy, and learning. *Journal of Research in Innovative Teaching & Learning*.

[21] Moran J., Briscoe G., Peglow S. (2018). Current technology in advancing medical education: perspectives for learning and providing care. *Academic Psychiatry*.

[22] Kauppi S., Muukkonen H., Suorsa T., Takala M. (2020). I still miss human contact, but this is more flexible—paradoxes in virtual learning interaction and multidisciplinary collaboration. *British Journal of Educational Technology*.

[23] Riva G., Mancuso V., Cavedoni S., Stramba-Badiale C. (2020). Virtual reality in neurorehabilitation: a review of its effects on multiple cognitive domains. *Expert Review of Medical Devices*.

